# Design of Semantic Matching Model of Folk Music in Occupational Therapy Based on Audio Emotion Analysis

**DOI:** 10.1155/2022/6841445

**Published:** 2022-06-18

**Authors:** Wensi Ouyang

**Affiliations:** School of Music Shaanxi Normal University, Xi'an Shaanxi 710119, China

## Abstract

The main semantic symbol systems for people to express their emotions include natural language and music. The analysis and establishment of semantic association between language and music is helpful to provide more accurate retrieval and recommendation services for text and music. Existing researches mainly focus on the surface symbolic features and association of natural language and music, which limits the performance and interpretability of applications based on semantic association of natural language and music. Emotion is the main meaning of music expression, and the semantic range of text expression includes emotion. In this paper, the semantic features of music are extracted from audio features, and the semantic matching model of audio emotion analysis is constructed to analyze ethnic music audio emotion through feature extraction ability of deep structure. The model is based on the framework of emotional semantic matching technology and realizes the emotional semantic matching of music fragments and words through semantic emotional recognition algorithm. Multiple experiments show that when *W* = 0.65, the recognition rate of multichannel fusion model is 88.42%, and the model can reasonably realize audio emotion analysis. When the spatial dimension of music data changes, the classification accuracy reaches the highest when the spatial dimension is 25. Analysing the semantic association of audio promotes the application of folk music in occupational therapy.

## 1. Introduction

Emotion analysis is to establish a harmonious man-machine environment by giving computers the ability to recognize, understand, express, and adapt to human emotions and make computers have higher and more comprehensive intelligence. Sentiment analysis is an important content of sentiment computing, and it is also a problem that must be solved in the field of sentiment computing. Music is the carrier of emotion and an important aspect of affective computing. In the emotional analysis of music, people usually like some sad music when they are sad and upset, in a happy mood, they like to listen to cheerful and dynamic music, and when they are calm, they tend to choose soothing and smooth light music, which is conducive to rationally solving problems and maintaining healthy psychology. These potential “emotional tendencies” can expand the corresponding emotions of music listeners, and these emotions will generate some “motivation” to solve the corresponding problems [1]. Filmmakers like to add background music to the movie to make the audience and the characters in the movie resonate and share a common mood, so that the audience can have a “good impression” on the movie. Music and emotion are inextricably linked. Music can affect emotions and also show emotions. Emotions can affect people's perception of music when they listen to songs. What makes music meaningful is the emotional connection between the participant and the listener. Emotion is the essential feature of music, and cognitive emotion has a corresponding relationship between acoustic vibration and nonsemantic structure of music. Music not only provides entertainment but also has many social and psychological applications. Emotion analysis has become one of the most active research fields in natural language processing. It has also been extensively studied in the fields of data mining [2], text mining [3], content recommendation [4], and information retrieval [5]. Because of its commercial value, academic value, and importance to society as a whole, sentiment analysis has expanded from computer science to other disciplines. The Internet has become an important medium for people to express their opinions and to get some information, and the information conveyed by others can influence our opinions. Therefore, an automatic sentiment analysis system is required, which usually contains sentiment classification modules. According to the different symbols, sentiment analysis can be divided into text sentiment analysis [6], video sentiment analysis [7], and audio sentiment analysis [8]. In the research of emotion recognition of audio, it mainly deals with the audio signal. The widely used audio features are: sound quality feature, spectrum feature, rhythm feature, and so on.

With the development of science and technology, the model has significantly enhanced the ability to extract effective features from a large number of data, and the topic of music therapy has attracted more and more people's attention. As music therapy workers, it is worth pondering and discussing to develop the cause of music therapy by using rich local music resources. The Chinese folk music culture is effectively applied to music therapy, and the Chinese folk music culture is carried forward through music therapy, so that it goes to the world. Guide the patient to sing, play, and write music for therapeutic purposes. The application of folk music culture to music therapy, effective music therapy internationalization of folk music culture, the development of music therapy with Chinese characteristics. Playing guqin cultivates the mind and forgets troubles, and the healer is completely immersed in music, which brings good practical results for occupational therapy. Folk music culture is broad and profound, with a long history, far-reaching connotations, and rich repertoire, which can express various artistic conceptions and feelings. To apply folk music culture into music therapy, one needs to know more about one's own music culture, and music therapy can be applied in a very wide range [9]. There are discrete model and dimensional model widely used in the field of music emotion cognition. The model includes four emotional adjectives, which are used to describe different emotional attributes in the music field and are classified into similar emotional types according to the categories. Each link in the emotional circle is connected with the left and right links in the emotional logic that there is a progressive relationship, and the progressive relationship represents the regular change of human emotions. The affective cluster of the affective ring, respectively, has been widely recognized and applied in the field of musical emotion analysis. The selection of emotion model depends on emotion recognition methods and specific application scenarios [10]. Emotional words in the model are extracted from people's perception of music and mainly consider the psychological feelings of listeners to the songs they listen to, which is in line with the actual situation of psychological interaction of musical emotions. But how to identify music nondescriptive query and music emotion analysis has become an important research topic for musicologists and psychologists.

## 2. Related Work

Musical emotion describes the inherent emotional expression of musical data, which is widely used in music retrieval, music understanding, and other music-related applications. Audio data is the most important form of music data expression, and a single note cannot show the beauty of music and cannot directly allow the composer and listener to carry out emotional communication, and it can be said that without audio, there is no music. Therefore, many researchers try to use audio processing to understand and analyze the emotion of music. Girgin proposed that music emotion classification based on audio data was an important method in music emotion analysis, which segmented audio data and extracted physical features. Lyrics are the important information of a song and the carrier of the content of the song, which most intuitively expresses that the content of the song is the original intention of the song [11]. Although social tags briefly contain users' understanding of the shared content, they are additional information about the semantic meaning of the shared content, which contains potential resource classification. Social tags can be applied to music field, including music classification of social tags, construction of semantic space, and other multiangle and multilevel applications. Juslin et al. proposed to use social labels of music resources to construct semantic space of music retrieval and use tag clustering to improve retrieval effect in tag space to obtain similar music [12]. If these tags can be well integrated into an application system, tag will play an important role in music information retrieval system. In music resource sharing website, social tag is the system user's understanding of music and emotional interpretation is the free gene of music.

Music develops with the development of human society, but music has timeliness. Music retrieval needs to express music in the form of music score according to the tempo and pitch of melody and search music data according to the similarity of melody. Gingras B. and others have provided four search means. Modern music retrieval system can process hundreds of millions of music data, but the new music retrieval system should pay more attention to the performance in online music retrieval, so that users from different social backgrounds can have a higher experience in retrieving music in different ways [13]. The content of music is very rich. It can be the rhythm of music melody or a piece of music. Content-based music information retrieval is a hot research topic at present. More and more online music retrieval systems use content-based music information retrieval technology. In the research of content-based music retrieval, humming retrieval is one of the main research directions. Vaidya and Kalita based their humming music retrieval on audio processing analysis and obtained the fundamental frequency distribution of input sound waves through autocorrelation measurement calculation [14]. Xu et al. proposed to extract audio features with an improved music melody contour extraction algorithm to remove the influence of noise brought by the environment and audio input equipment on the humming query [15]. Pandeya and Lee proposed the method of extracting feature kernel for semantic music retrieval, combined audio information and social context information for semantic music information retrieval, and developed the corresponding music retrieval system based on semantic understanding [16]. Based on the rhythm and timbre of music, Belyk et al. constructed a multilabel emotion recognition model based on principal component analysis, extracted audio features through multilevel convolutional network, and learned the vector representation of music labels for automatic music labelling [17]. Traditional music retrieval methods cannot meet the needs, so we need to find new music retrieval methods and ways. With more and more resources on the Internet, automatic text classification by computer is an important research topic of natural language processing and artificial intelligence. Related research is still in the stage, related technology is still to be improved, and it is difficult to analyze music features and immature representation of music, which affects the extraction of music features.

The main method of the audio model based on emotional semantic matching proposed in this paper is to describe the audio in the emotional semantic space and then identify and match the audio through the emotional semantic, so as to give the music list that best meets its emotional demands in occupational therapy.

## 3. Semantic Matching Model of Folk Music Based on Audio Emotion Analysis

### 3.1. Feature Extraction of Ethnic Music Audio

The automated description of music content is based on the feature extraction of computable time-frequency domain signals. The concept and extraction process of each feature will be described below. Frequency is a simple sine curve defined as the number of cycles per second, or Hertz (Hz). For example, a sine wave has a frequency of 440 Hz, or 440 cycles per second. The reciprocal of frequency is the period, and the physical meaning is the number of seconds, that is, the time interval of sinusoidal signal in a oscillation period [18]. In the time domain, the analogy signal is sampled once every second to obtain the data signal. The spectrum diagram of the time domain signal is the expression of the audio signal in the frequency domain. The spectrum diagram of the signal can be obtained by Fourier transform, and the result value of Fourier transform is usually expressed by amplitude and phase, as shown in Figure 1.

The figure shows the corresponding frequency-domain features of musical notes played by instruments. All sound frequency positions are the same. Spectrum is an important factor determining sound quality or timbre. Complex sounds contain relevant amplitude signals of different frequencies. For the sampled signal, compute the discrete Fourier transform. Frequency spectrum analysis of audio signals is usually carried out on a short segment, called a “frame,” by which the short-time Fourier transform can capture the frequency content changes in time. The mathematical expression of this transformation is the addition of a window function to the discrete signal, which is generally bell shaped and stationary over a short period of time.

### 3.2. Semantic Emotion Recognition Algorithm

In this study, the feature extraction of speech emotion recognition algorithm and the learning method of training model are used for recognition, as well as the calculation and judgment of speech emotion recognition through the query of emotion dictionary combined with sentence structure. When semantic understanding is carried out through emotion dictionary query, it is necessary to establish an emotion dictionary library to obtain the annotation value of emotion. In this paper, some famous emotion dictionaries are sorted out to establish the emotion dictionary library. In this paper, the dictionary of negative words used in this paper is constructed by selecting common negative word dictionaries and adding popular negative descriptions on the Internet. Emotion recognition is carried out by querying the emotion dictionary, and emotion words and judgment words are marked with familiar words, and adverbs of degree are marked numerically. Different emotional words represent different emotional tendencies and sizes, so their annotations are also different. Different degree adverbs have different functions and degrees, so determining the value of degree adverbs is also an important part in the process of emotion recognition [18]. In the process of emotion recognition, adverbs of degree need to be marked numerically. Through the modification of adverbs of degree, the intensity of emotion will also change.

In this paper, degree adverbs are divided into four grades, and then by setting different emotional weights for each degree adverb, degree words can modify the following emotional words through this processing. By sorting out and processing the emotion word dictionary, degree word dictionary, and negative word dictionary, this paper builds an emotion dictionary base of common words on the basis of previous studies, which can be used for text emotion recognition in the future. Affective orientation is the value of the valence direction in the dimensional coordinate emotion model, which represents an emotional orientation and represents the parameters of the positive and negative emotions and the positive and negative degrees of the parties. The semantic emotion recognition system based on emotion dictionary is quick to construct, with good recognition effect and fast recognition speed [19]. The proposed sentiment analysis algorithm is mainly composed of text cutting and conversion, sentiment location, and sentiment aggregation. After obtaining the text information, the text information needs to be converted into text cutting first, and the sentence is split into word sets. Text slice transformation is the basis of text information processing; emotion recognition technology cannot do without text slice transformation. Through the study of Chinese natural language processing, text cutting conversion uses language rules to find the separation between words and their own words and mark the parts of speech. Only through the multichannel fusion of multidomain knowledge can we do a good job of word segmentation.

### 3.3. Semantic Matching Technology Framework Based on Audio Emotion Analysis

In music retrieval, feature selection, representation, and matching are the core techniques. Based on the research and analysis of music physical and perceptual characteristics, this paper takes melody as the main feature and establishes melody representation model through pitch extraction and dynamic threshold segmentation algorithm to retrieve music data sets and input music samples. In order to improve the retrieval accuracy, genetic algorithm was used to align the template and correct the individual difference of matching input. The fusion Euclidean distance and similarity measure matching template is applied to enhance fault tolerance and generalization ability. Finally, the effectiveness of the algorithm is verified by prototype system. Musical features can be roughly divided into three levels—physical features, acoustic features, and perceptual features. The semantic matching technical framework based on audio sentiment analysis is shown in Figure 2. Physical features mainly refer to the audio content recorded by physical carriers in a certain format, which is presented in the form of streaming media. Acoustic level features mainly include time and frequency domain features, such as pitch frequency, short-term energy, zero crossing rate, LPC coefficient, and MFCC coefficient, which are the performance characteristics of audio itself and are often used in each stage of speech recognition. Perceptual characteristics reflect people's descriptions of music feelings, such as pitch, rhythm, tone strength, and timbre. Perceptual characteristics can usually be extracted from physical characteristics, and it is more consistent with human recognition and judgment of music content.

Music is a discrete sequence of notes that changes over time, yet feels like a complete entity of notes that change over time. The melody contour of music is the characteristic of pitch changes with time, and pitch is determined by the pitch frequency of music. Therefore, melody contour can be extracted and described by extracting pitch and describing pitch with appropriate model. This paper proposes a melody representation model based on the standard template and input template, extracts the pitch template of the audio file input by the user from the chord music file, and establishes the relationship between the standard pitch frequency templates, because these two templates belong to the category of pitch frequency, and their appearance is similar after normalization. On the basis of the above research, the melody representation model is further improved, and the appropriate matching algorithm is proposed to match the final retrieval results.

### 3.4. Construction of Semantic and Audio Emotion Recognition Model

The model uses prosodic feature, spectral feature, voice quality, and audio feature to carry out emotion recognition. With the development of speech denoising technology, the accuracy of speech recognition has been improved. The text recognized by speech has strong credibility, and the semantic recognition by querying the dictionary can ultimately preliminarily determine the semantic emotional state of speech information [20]. This paper establishes a speech emotion recognition system combining semantics, and the overall system structure is shown in Figure 3. Phonetic features have a high recognition rate in emotional intensity, but there is a certain limitation in the identification of emotional orientation. Semantic emotion recognition, on the other hand, has a very good performance in identifying emotional tendencies. Semantic combination of speech emotion recognition model is set up, respectively, to identify the text emotion tendentiousness and voice acoustic characteristics described in the emotional tendency and active situation, and then, the text recognition tendency and acoustic characteristics identification of multimodal integration level of emotional tendency to make decisions get a multimodal fusion after emotional tendencies. The multichannel fusion process of text emotion recognition and acoustic emotion recognition will be carried out in the judgment of emotion orientation, namely, the valence axis in the dimensional emotion model.

This gap is a relatively small difference in emotion recognition. When prosodic features are difficult to identify the positive emotion, the method of believing the text emotion orientation is adopted to adjust the emotion value [21], and the emotional tendency of the speech channel and the text channel is identified. The output data of speech channel are the result of recognition, the probability of positive emotional orientation, and the probability of negative emotional orientation. The output data of the text channel is the affective tendency value obtained through calculation. The two channel results of the model are used as input signals to the final model. The decision level fusion model is used to fuse the two recognition results. Finally, the recognition and classification of discrete emotion model based on semantic combination is realized.

### 3.5. Feature Model Training

This design sets up a four-layer model, based on the model, respectively, using audio features and lyric features to classify emotions. The input layer in the network model is set as 100 and 130 nodes, respectively, according to the characteristic dimension of the input, and the learning rate is initialized as 0.05. The number of nodes in the hidden layer compresses the data layer by layer, and the number of nodes in the hidden layer is 400, 200, and 150, and the number of iterations is 150. The SoftMax layer at the end of the network structure takes the emotional category of music as the output, with a total of 4 categories, so the number of nodes in the output layer is set to 4.

Figure 4 shows the influence of iteration times on matching error during network model training. By analysing the above figure, it can be clearly obtained that the relationship between the number of iterations and the matching error is that the latter gradually decreases with the increase of the former. When the number of iterations increases from 1 to 100, the classification error decreases rapidly. When the number of iterations increases to 150 to 200, the variation of classification error is no longer obvious. On the other hand, it can be concluded that the feature extraction ability of deep confidence network with deep structure is stronger than that of shallow network.

## 4. Experimental Results and Analysis

The music samples in this paper are from 1200 songs in the database, 1000 of which are used as training samples and the remaining 200 as test samples. The emotions of the sample songs were divided into 6 categories: excitement, sadness, fear, anxiety, relaxation, and joy. The audio was in a unified format, and 30 s of music fragments with the most emotional representation were selected for the classification of musical emotions. One thousand songs were randomly divided into five groups, and then, the five groups were trained separately.

### 4.1. Recognition Rate of Semantic Matching Model

The experimental training set carries out multichannel fusion of the two sets of data. In the recognition process, the recognition results of the speech channel need to be processed first and converted into the data that can be used as the input of multichannel fusion, which is converted into

(1) $$\begin{array}{c} W_{v}=P_{p}-P_{n}, \end{array}$$

where *W*_*v*_ is voice channel input, *P*_*p*_ is the probability that speech recognition results tend to be positive, and *P*_*n*_ is the speech recognition results that tend to be the negative probability.

The output of this formula is a value from minus one to one, and the output of the text channel is also processed accordingly. By multiplying the result of text emotion recognition by a smaller weight, it is converted into the input data of the text channel and transformed into

(2) $$\begin{array}{c} W_{s}=0.02\times A_{s}, \end{array}$$

where *W*_*s*_ in the text channel input; *A*_*s*_ is the sentence emotion value. In this way, text channel input and voice channel input are transformed to the same data format and order of magnitude, and then, the weighted multichannel fusion is carried out for the two groups of data. The calculation of multichannel fusion channel is obtained by

(3) $$\begin{array}{c} W_{e}={\frac{W}{W}}_{s}+\frac{W_{v}}{1-w}. \end{array}$$

In the formula, we output multichannel fusion results; *W*_*e*_ is the weight of text channel input in the weighted multichannel fusion process, *W*_*s*_ is the text channel input, and WV is the voice channel input.

Finally, the positive and negative values are used to judge the emotion recognition result after multichannel fusion. By adjusting different weights, the recognition rate of each weight is counted, and the weight with the best recognition result is selected as the parameter of the multichannel fusion channel of the multichannel model.  Figure 5 shows the recognition rate when different weights *W* are selected in the semantic matching model.

According to the figure, when *W* =0.65, the best recognition rate obtained by the multichannel fusion model is 88.4.2%. Under the optimal parameters, the recognition rate of emotion, sadness, fear, anxiety, ease, and joy is 80.3%, 82.6%, 87.5%, 83.4%, 81.2%, and 88.4%, respectively. The semantically integrated speech emotion recognition experiment finally locates each sample to each specific emotion by combining the recognition results of the activation coordinate axis of each sample and the recognition results of the multichannel emotion orientation. The matching recognition rate was 85.3%, 82.5%, 80.3%, 79.5%, 76.2%, and 81.4%, respectively.

### 4.2. Evaluation of Audio Spatial Feature Vectors

The method of graph learning is used to make a series of spatial feature vectors and original feature vectors by integrating audio and text information, which proves the validity of the musical space representation. In the original space, due to the heterogeneity between different modal features, in the graph learning method, the test samples of each mode can only search for training samples in their own space, while the spatial representation method can make the test samples search for modes. The classification accuracy of spatial learning methods is shown in Figure 6.

It can be seen from the figure that the classification accuracy of using spatial features is better than that of original spatial features in most classes, which proves the validity of spatial features. This validity is precisely because spatial features make better use of the correlation between modal data than original spatial features. When the spatial dimension of music data changes, the classification accuracy reaches the highest when the spatial dimension is 25. It can be seen from *W* that these two curves do not have the change rule of Ming Si. Such irregularity of single mode and result improvement in multimode fusion indirectly prove the effectiveness of spatial representation in describing the correlation between modes.

### 4.3. Ability to Identify Emotional Tendencies

The audio in the data set is uniformly converted into WAV format. Each song has a long audio time and often has the same music melody. Therefore, 30 music clips of 15-45 seconds per song were used as audio data for emotional classification. Since all the audio files in the data set cannot be directly input as training data, it is necessary to extract representative music features from the audio files. The accuracy of audio emotion construction and the coverage of emotion will affect the result of emotion analysis. In different scenarios, the effect of audio sentiment analysis may not be as expected. The main purpose of the experiment is to verify the ability of the proposed music retrieval model based on affective semantic relevance to solve the problem of nondescriptive music query processing in music retrieval system, in order to verify the influence of different music matching methods on model recognition ability. The verification of the combined emotion recognition system is achieved by comparing the experimental results obtained from three experiments, namely, the emotion recognition based on voice acoustic features and the speech emotion recognition based on text emotion recognition and semantic combination. The experimental results and data of the three experiments are shown in Figure 7.

The data in the graph is expressed in the form of matrix graph, and the recognition rate of the three emotion recognition algorithms can be seen intuitively. The recognition accuracy of traditional support vector machine can be improved slightly by dimensional-classification recognition method. On this basis, the recognition rate can be improved significantly by combining semantic recognition results with multichannel fusion. Among them, the recognition rate of anxiety and fear with low activity increased greatly, indicating that there is some complementarity between text information and phonological features in emotion recognition.

### 4.4. Emotional Semantic Matching Accuracy

Accuracy rate and recall rate were used as evaluation indexes. Accuracy is the number of correctly matched words divided by the total number of verified data. Precision is the ratio of the number of correctly matched topics to the number of topics judged by the model. The recall rate is the ratio of the number of correctly matched topics to the number of topics that belong to that topic. Recall rate formula is as follows:

(4) $$\begin{array}{c} \text{R}=\frac{\text{A}}{\text{A}+\text{C}}. \end{array}$$

When random bars were selected as music units in the experiment, the reason why the two emotional themes of sadness and joy were selected in the experiment was that they had higher emotional differentiation. Compared with the experimental results without emotion screening, the experimental results are significantly improved, especially the effective information in the sequence can be better captured. Module and attention mechanism are effective in extracting sequence features. After training, they can effectively distinguish different emotions and are less affected by the intensity of emotions. According to the experimental results, the music climax segment is selected as the adaptive matching effect of the music unit validation model, and the experimental results are shown in Figure 8.

Figure can be seen that using highlights data model in 6 emotional subject adaptability experiment accuracy is over 75%, in sadness and joy these two emotions obviously on the theme of the accuracy of more than 82%, therefore, although the model has certain accuracy, but on the whole model can be done more effectively music clips and words to match. The matching effect of excitement and ease is better, and the accuracy rate is 83.35% and 84.81%, respectively. The matching effect of emotional anxiety is poor, and both emotional focus and fear need to be improved. It performs best in the results of emotional semantic matching between music and text. Audio features can describe the audio features of songs more effectively, and the feature vector model has higher accuracy and the best analysis effect.

## 5. Conclusion

With the development of the Internet, folk music retrieval is not limited to text retrieval, but music retrieval through the audio information of songs. Based on the music audio signal characteristic, the essential characteristics extracted from folk songs of audio data, using artificial extraction sequence characteristics as the training data and semantic matching algorithm, the proposed songs build audio semantic matching model of sentiment analysis, and on this basis, the matching accuracy is used to identify the semantic combination of research and finally prove the feasibility and advantage of research results. In the process of participating in the establishment of emotional speech database, through the analysis of annotation data, the potential relationship between emotion types and dimension coordinates is summarized, so that the expression of emotion can be more detailed and comprehensive, and the changing trend of emotion can be better reflected. By identifying the transformation model for training, the data amount of training set corresponding to the training speed is increased effectively. The recognition accuracy of traditional support vector machine can be improved slightly by dimensional-classification recognition method. On this basis, the recognition rate can be improved significantly by combining semantic recognition results with multichannel fusion. However, there are some limitations in the research process, and further research is still needed in music classification. Emotion recognition technology has a wide range of application scenarios, many fields have extremely important influence and demand, and has great research value. In the future, I will continue to improve the semantic matching model and study the influence of emotional cognition on music retrieval system.

## Figures and Tables

**Figure 1:** Spectrum diagram of the dispersion music signal.

**Figure 2:** Semantic matching technology framework based on audio sentiment analysis.

**Figure 3:** Structure diagram of speech emotion recognition system with semantic combination.

**Figure 4:** Network model training iteration error graph.

**Figure 5:** Graph of recognition rate of semantic matching model.

**Figure 6:** Statistical chart of accuracy of audio space feature vector analysis.

**Figure 7:** Semantic matching speech emotion recognition experimental results data graph.

**Figure 8:** Adaptive matching effect of music unit validation model.

## Data Availability

The data used to support the findings of this study are available from the corresponding author upon request.
